# Analysis of Clinical Outcomes of Different Fertilization Methods in Patients with ≤3 Eggs Retrieved

**DOI:** 10.1155/2022/9467568

**Published:** 2022-03-16

**Authors:** Shuang Wang, Xiaoyan Zhang, Hongchu Bao, Yuanqing Cui

**Affiliations:** Department of Reproductive Medicine, Qingdao University Affiliated Yantai Yuhuangding Hospital, Yantai, Shangdong 264000, China

## Abstract

**Objective:**

To explore the intracytoplasmic sperm injection (ICSI) and *in vitro* fertilization (IVF) method on the clinical outcomes of infertile women with ≤3 eggs retrieved. *Study Design.* We retrospectively analyzed a cohort of female patients who received IVF/ICSI to assist pregnancy with retrieved eggs ≤3. The general conditions, i.e., two pronuclei (2PN) fertilization rate, abnormal fertilization rate, high-quality embryo rate, cycle cancellation rate, pregnancy rate of fresh embryo transfer, cumulative pregnancy rate, and miscarriage were compared between the two groups.

**Results:**

When the number of retrieved eggs was one, the fertilization rate of 2PN was higher and the cycle cancellation rate was lower in the ICSI group than in the IVF group (*P* < 0.05). The pregnancy rates of fresh embryo transfer, frozen-thawed embryo transfer, and the cumulative pregnancy rate were all higher in the ICSI group than in the IVF group (*P* < 0.05). When the number of retrieved eggs was two, the pregnancy rate of frozen-thawed embryo transfer and cumulative pregnancy rate in the ICSI group were higher than those in the IVF group (*P* < 0.05). When the number of retrieved eggs was three, the fertilization rate of 2PN and the pregnancy rate of frozen-thawed embryo transfer were higher in the ICSI group than those in the IVF group (all (*P* < 0.05)).

**Conclusions:**

For patients with one egg retrieved, ICSI fertilization can reduce abnormal fertilization rate and cycle cancellation rate and improve cumulative pregnancy rate significantly enhancing patients' benefits. However, increasing the number of eggs retrieved decreases the advantages of ICSI fertilization.

## 1. Introduction

With the development of assisted reproductive technology (ART), the clinical pregnancy rate has gradually increased. Studies have shown that the clinical pregnancy rate increases with the number of retrieved eggs [1, 2]. However, patients with decreased ovarian reserve function and low ovarian response have fewer eggs retrieved in a single operation, which is often less than or equal to 3. In these patients, fewer embryos can be transferred and the pregnancy rate is low [3]. Multiple egg retrieval operations are needed to achieve a successful pregnancy ultimately increasing the trauma of patients [4]. At present, the problem that needs to be solved is to improve the effective utilization of eggs when the number of eggs retrieved is low. An effective approach is to reduce the occurrence of abnormal fertilization, such as the occurrence of fertilization failure (zero pronucleus, 0PN) and multiple pronuclei (multi-PN, MPN) [5].

Intracytoplasmic sperm injection (ICSI) technology has been applied to non-male-derived infertility in the world, such as preimplantation genetic testing, failure of more than two ART assisted pregnancies, less than 5 eggs retrieved, patients ≥38 years old, and unexplained infertility [6]. The National Assisted Reproductive Technology Surveillance System (NASS) reported that the utilization rate of ICSI for male infertility had increased from 76.3% to 93.93% between 1996 and 2012. The utilization rate of ICSI in nonmale factor caused infertility had increased from 15.4% to 66.9% [7]. However, since ICSI is an invasive procedure, experts have different opinions on whether ICSI should be applied to patients with fewer eggs retrieved [8, 9]. In China, ICSI indications are relatively strictly controlled, and the increase of ICSI application rate is not as significant as that in Western countries. Scientists have discussed for many years whether ICSI indications should be extended to low retrieved egg number, poor fertilization history, and unexplained infertility. However, the conclusions remain controversial [10]. For the pregnancy outcome of patients with retrieved eggs ≤3, some studies suggest that ICSI can reduce the abnormal fertilization rate and cycle cancellation rate and improve the number of transferrable embryos and pregnancy rate [11, 12]. Other studies suggest that ICSI and IVF have no difference in pregnancy outcomes [13, 14]. Therefore, we retrospectively analyzed patients with retrieved egg number ≤3 and divided them into an ICSI group and an IVF group according to different fertilization methods they received. We matched the patients in the two groups based on age and ovulation induction scheme to reduce selection bias. By comparing the mature egg (MII) rate, 2PN fertilization rate, abnormal fertilization rate, high-quality embryo rate, cycle cancellation rate, pregnancy rate of fresh embryo transfer, miscarriage rate, cumulative pregnancy rate, and cumulative miscarriage rate, we investigated the effects of ICSI and IVF on the pregnancy outcomes of patients with retrieved eggs ≤3.

## 2. Materials and Methods

### 2.1. Research Subjects

This study was approved by the Ethics Committee of Qingdao University-affiliated Yantai Yuhuangding Hospital. All patients signed IVF or ICSI informed consent forms. Infertility patients who received IVF/ICSI in the Department of Reproductive Medicine, Qingdao University-affiliated Yantai Yuhuangding Hospital between January 2017 and June 2020 were selected for this study. Patients' inclusion was based on the following: (1) ≤3 retrieved eggs; (2) no abnormality in uterus and hysteroscopy showed that the endometrium was normal; (3) pituitary prolactin (PRL) was within normal range (6.0 ng/ml 29.9 ng/ml); and (4) normal thyroid function. Patients with (1) 42 years of age or above; (2) suffering from diabetes, hypertension, or other uncontrolled medical complications; and (3) received preimplantation genetic testing (PGT) were excluded from this study.

## 3. Research Methods

### 3.1. Grouping

The patients were divided into an ICSI group and an IVF group according to the different fertilization methods they received. After screening by inclusion and exclusion criteria, 326 cycles were included in the ICSI group, and 2,086 cycles that had ≤3 retrieved eggs were included in the IVF group.

### 3.2. Ovulation Induction Process

Ovulation induction treatment included microstimulation treatment, antagonist treatment, and natural cycle IVF.

- Microstimulation treatment: on the second day of the menstrual cycle, letrozole (0.5 mg/tablet, Furui, Hengrui Medicine, China) was given orally at 5 mg/d for 5 days After five days of letrozole treatment, urinary follicle stimulating hormone (75 IU/package, Lishenbao, Lizhu Medicine, China) for injection was initiated. The initial dose was 150–300 IU/d and continued until the day of HCG.
- Antagonist treatment: on the second day of menstrual cycle, recombinant human follicle stimulating hormone (rFSH, 600 IU/package, Puregon, Organon, the Netherlands) was injected daily. The initial dose was 150–300 IU/d, and the dosage was adjusted according to the patient's condition until the maximum follicle diameter was 12 mm or *E*_2_ level was higher than 1,468 pmol/L. Subsequently, GnRH antagonist (Ganirelix, 0.25 mg/package, MSD, USA) 0.25 mg/d was added to the treatment schedule until the day of HCG.

Follicular development was monitored by transvaginal ultrasound. When the diameter of at least one or two follicles was ≥1.8 cm, human chorionic gonadotrophin (hCG, 2,000 IU/package, Lizhu, Zhuhai, China) at 6,000 IU was injected subcutaneously to the patient. After 36 h, ultrasound-guided transvaginal egg retrieval was performed.

### 3.3. Fertilization and Embryo Transfer

IVF or ICSI was used according to the quality of semen. In IVF, 50 ul microdrop insemination technique was used. Sperm at the insemination concentration of 10,000 sperm/50 ul was added into the microdrop in insemination dish using a Pasteur pipette, and one oocyte was added to each microdrop. Before ICSI insemination, oocytes were degranulated. MII-stage oocytes were selected for ICSI insemination. After immobilization, the sperm was aspirated into an injection needle so that the sperm head was located at the tip of the injection needle. The tip of the needle was moved into the droplet containing an oocyte. The oocyte was fixed with the fix needle so that the first polar body was located at 11–12 o'clock position or 6 o'clock position. Next, the injection needle passed through the zona pellucida and entered the cytoplasm of the oocyte. After the oocyte membrane was broken, the sperm was slowly injected into the central area of the oocyte, and then, the injection needle was slowly withdrawn.

On the third day after oocyte retrieval, one or two embryos were transferred to the uterine cavity of the patient and the remaining embryos were cryopreserved. After embryo transfer, progesterone soft capsule (Utrogestan, 100 mg/capsule, Laboratoires Besins International, France) at 200 mg was given intravaginally, once every 8 h for luteal support. On the 14^th^ day following embryo transfer, hCG levels of the patients were determined. The level of hCG >5.0 IU/L was considered biochemical pregnancy. On the 35^th^ day after the embryo transfer, patients received ultrasonography, the appearance of the gestational sac confirmed clinical pregnancy. For frozen-thawed embryo transfer (FET), patients with regular menstrual cycle were treated with natural cycle plan for endometrial preparation, while patients with irregular menstrual cycles were treated with hormone replacement plan for endometrial preparation. The embryo transfer criterium was based on that the endometrium should be ≥8 mm with homogeneous echo.

### 3.4. Observation Index

The general conditions of the patients, including age, duration of infertility, type of infertility (primary/secondary), basic FSH, basic *E*_2_, BMI, AMH, ovulation induction scheme, and abnormal semen of the male were observed. Laboratory and clinical outcomes were recorded, including MII rate (number of mature eggs/number of retrieved eggs), 2PN fertilization rate (2PN fertilized eggs/number of mature eggs), fertilization failure rate (number of mature eggs−number of 2PN fertilized eggs/number of mature eggs), high-quality embryo rate (number of high-quality embryos/number of 2PN cleaved embryos), cycle cancellation rate, pregnancy rate and miscarriage rate of fresh embryo transfer, pregnancy rate and miscarriage rate of frozen-thawed embryo transfer, miscarriage rate, and cumulative pregnancy rate. In this study, normal fertilization was defined as zygotes with 2PN following ICSI or IVF. Fertilization failure was defined as zero oocytes reaching the zygote stage with 2PN. The cycle cancellation rate only referred to the cycle cancelled due to the absence of transferrable embryos because of the failure of fertilization. The cumulative pregnancy rate referred to the total number of pregnancies achieved in all egg retrieval cycles analyzed in this study with normally fertilized embryos following fresh embryo transfer and frozen-thawed embryo transfer.

### 3.5. Statistical Analysis

The statistical software package (SPSS 20.0) was employed for statistical processing and analysis. Mean ± standard deviation (‾x ± *s*) was used for expressing measurement data, while percentage (%) was used for expressing count data. The analysis of the measurement data was carried out using independent sample *t*-test, while Fisher exact test and chi-square test were employed for the analysis of count data. (*P* < 0.05) was considered statistically significant.

## 4. Results

### 4.1. Comparison of General Data between the ICSI Group and IVF Group

After screening using inclusion and exclusion criteria, there were 326 cycles in the ICSI group and 2,086 cycles in the IVF group. There were no significant differences in age, infertility duration, body mass index (BMI), basic *E*_2_, AMH, and ovulation induction scheme between the two groups with (*P* > 0.05) suggesting that the two groups were similar in terms of basic characteristics. However, the proportion of primary infertility was higher in the ICSI group than that in the IVF group (*P* < 0.05). The basic FSH value was higher in the ICSI group than that in the IVF group (*P* < 0.05). The proportion of abnormal semen of males in the ICSI group was also higher than that in the IVF group (*P* < 0.05). The details of patients' demographics and other characteristics are shown in Table 1.

### 4.2. Comparison of the Clinical Outcomes between the ICSI Group and IVF Group When ≤3 Eggs Were Retrieved

The fertilization rate of 2PN was higher in the ICSI group than that in the IVF group (*P* < 0.05). The cycle cancellation rate was markedly higher in the IVF group than that in the ICSI group (*P* < 0.05). The pregnancy rate and cumulative pregnancy rate were both higher in the ICSI group than that in the IVF group ((*P* < 0.05), Table 2).

### 4.3. Comparison between the ICSI Group and IVF Group When the Number of Retrieved Eggs Were One, Two, and Three, Respectively

When the number of retrieved eggs was one, the fertilization rate of 2PN was higher in the ICSI group than that in the IVF group (*P* < 0.05). The cycle cancellation rate was higher in the IVF group than that in the ICSI group (*P* < 0.05). The pregnancy rates of fresh embryo transfer and frozen-thawed embryo transfer as well as cumulative pregnancy rate were all significantly higher in the ICSI group than that in the IVF group (*P* < 0.05).

When the number of retrieved eggs was two, the pregnancy rate of frozen-thawed embryo transfer and cumulative pregnancy rate were higher in the ICSI group than that in the IVF group (*P* < 0.05).

When the number of retrieved eggs was three, the fertilization rate of 2PN was significantly higher in the ICSI group than that in the IVF group (*P* < 0.05). The pregnancy rate of frozen-thawed embryo transfer was higher in the ICSI group than in the IVF group (*P* < 0.05). Detailed comparison between the groups is shown in Table 3.

## 5. Discussion

In the IVF cycle, if all or most of the eggs are not fertilized or fertilized abnormally and there is no transferrable embryo, it will bring a double blow to the patient economically and mentally [15]. The key to successful pregnancy for patients with ≤3 eggs retrieved is to obtain as many transferrable embryos as possible. The premise of obtaining transferrable embryo is to obtain normally fertilized embryo. Most of the patients whose number of retrieved eggs is ≤3 have poor ovarian function and low ovarian response. Studies have shown that the live birth rate in patients with poor ovarian function decreases. However, with the increase of the number of retrieved eggs, the cumulative live birth rate increases. At the same time, the proportion of cycles cancellation due to the lack of transferrable embryos decreases significantly [1]. Patients with ovarian dysfunction and low ovarian response often need multiple egg retrieval to achieve pregnancy. Multiple egg retrieval operations can cause enormous physical and psychological trauma and economic burden to the patients. How to improve the effective utilization of retrieved eggs and increase the pregnancy rate of patients with ≤3 retrieved eggs was the focus of this study.

According to the statistics of 2,414 cycles, the proportion of primary infertility was higher in the ICSI group than that in the IVF group. This is because the proportion of poor semen quality in the ICSI group was higher than that in the IVF group, and the proportion of infertility caused by male factors was also higher in the ICSI group. The basic FSH value in ICSI group was higher than that in the IVF group (11.49 ± 5.89 vs 10.55 ± 76) (*P* < 0.05). However, the number of eggs retrieved in enrolled patients was fixed, and there was no statistical difference in ovulation induction treatment and AMH value. Therefore, the basic FSH value had no impact on this study. The basic FSH values of the two groups were both higher than 10 IU/L, and the AMH values were both less than 1 ng/ml, suggesting that the ovarian reserve function was decreased in both groups.

In this study, in patients with ≤3 eggs retrieved, the 2PN fertilization rate was higher in the ICSI group than that in the IVF group (*P* < 0.05), while the cycle cancellation rate was higher in the IVF group than in the ICSI group (*P* < 0.05). The pregnancy rate of frozen-thawed embryo transfer and cumulative pregnancy rate were both higher in the ICSI group than in the IVF group (*P* < 0.05). However, after further grouping patients according to the number of retrieved eggs (one, two, and three), we found when the number of retrieved eggs was one that the pregnancy rates of fresh embryo transfer and frozen-thawed embryo transfer, and the cumulative pregnancy rate were all higher in the ICSI group than that in the IVF group (*P* < 0.05). When the number of retrieved eggs was two, the pregnancy rate of frozen-thawed embryo transfer and cumulative pregnancy rate of the ICSI group were higher than those of the IVF group (*P* < 0.05). When the number of retrieved eggs was three, the pregnancy rate of frozen-thawed embryo transfer in the ICSI group was higher than that of the IVF group (*P* < 0.05). Cycle cancellation can be caused by many reasons, including luteal phase ovulation induction, thin endometrium, and abnormal fertilization. Therefore, abnormal fertilization-caused cycle cancellation should be analyzed separately to reflect the difference of clinical outcomes caused by different fertilization methods. In this study, in patients with one egg retrieved, 22.87% (177 cycles) of IVF group patients and 14.29% (17 cycles) of the ICSI group patients were cancelled due to abnormal fertilization. The patients who had no transferrable embryos due to abnormal fertilization needed to receive another ovulation induction and egg retrieval operation. The patients who have less transferrable embryos due to abnormal fertilization will lose the chance of frozen-thawed embryo transfer, which will reduce the cumulative pregnancy rate. It suggested that ICSI is a better fertilization method for patients with one egg retrieved.

In general, ICSI is more beneficial than IVF in patients with one egg retrieved when compared with patients with two or three eggs retrieved. It not only can improve the cumulative pregnancy rate and reduce the cycle cancellation rate but also can reduce the potential risk and trauma of multiple egg retrieval operations. In previous studies, whether ICSI can improve the pregnancy outcome of patients with ≤3 eggs retrieved remains controversial. Some researchers believe that ICSI can improve the number of transferrable embryos and the pregnancy rate [11, 12]. Some others consider that compared with IVF, ICSI has no significant impact on pregnancy outcome [13, 14]. In previous studies, it may be because the number of cycles with one, two, and three eggs retrieved was not consistent, e.g., there were more patients in the group with one egg retrieved. ICSI can provide more transferrable embryos and improve the cumulative pregnancy rate. ICSI can improve pregnancy outcome. In contrast, when most patients had 2 or ≥3 eggs retrieved, ICSI-provided improvement of pregnancy outcome was limited, which may be the reason for inconsistent statistical outcomes.

According to literature reports, in women with advanced age and nonmale factor infertility, ICSI does not significantly improve the embryo quality and clinical outcomes [16, 17]. Our study indicated that in patients with nonmale infertility, advanced age is not a criterion for whether choose ICSI as *in vitro* fertilization method. Patients with advanced ages can also obtain more than three embryos. Low number of retrieved eggs is the criterion for ICSI fertilization.

The damage of ICSI to oocytes remains controversial, and there is no clear evidence to show that ICSI can affect the health of offspring [18, 19]. In our study, when patients with ≤3 eggs retrieved, high-quality embryo rate was 56.70% in the ICSI group and 56.74% in the IVF group. There was no significant difference between the two groups. This result suggests that ICSI does not damage the quality of embryo. The miscarriage rate of fresh embryo transfer was 13.33% in the ICSI group and 15.17% in the IVF group, with no significant difference between the two groups. Regarding frozen-thawed embryo transfer, the miscarriage rate in the ICSI group and IVF group was 14.61% and 10.16%, respectively, with no significant difference between the two groups. The cumulative miscarriage rates were also similar between the two groups (14.29% in the ICSI group vs. 13.07% in the IVF group). These data suggest that ICSI does not increase the miscarriage rate. We will continue to track the impact of ICSI on the health of offspring.

The limitations of this study are as follows: (1) The difference between groups was not completely eliminated, especially the semen quality of the male, which is also a factor affecting the quality of pregnancy. Our next study is to use the randomized controlled trial (RCT) method to group patients to eliminate selection bias. (2) The dataset analyzed in this study was from a single center. Thus, the data are of limitation. The analytic results cannot represent the overall situation. However, our findings still provide a reference for clinical practice.

## 6. Conclusion

Patients with ovarian dysfunction and low ovarian response often need multiple egg retrieval to achieve pregnancy causing enormous physical and psychological trauma and economic burden to the patients. This study focused on the comparison of ICSI and IVF as effective utilization of retrieved eggs and increasing the pregnancy rate of patients with ≤3 retrieved eggs. Results of this study results show that for infertility patients with ≤3 eggs retrieved, ICSI can improve the normal fertilization rate and reduce the cycle cancellation rate caused by fertilization failure. In particular, for patients with one egg retrieved, the benefits of one egg retrieval cycle can be maximized so as to reduce the trauma and complications caused by multiple egg retrieval operations. However, with increased number of eggs retrieved, the advantages of ICSI fertilization decrease.

## Figures and Tables

**Table 1:** Comparison of the general data between the ICSI group and IVF group.

Index	ICSI group *n* = 326	IVF group *n* = 2086	F/*x*^2^	*P* value
Age (years, ‾x ± *s*)	34.88 ± 3.82	35.11 ± 4.03	1.248	0.348
Duration of infertility (years, ‾x ± *s*)	4.97 ± 3.35	4.80 ± 3.56	0.866	0.395
Infertility			8.050	0.005
Primary infertility (case (%))	175 (53.68)	944 (45.25)		
Secondary infertility (case (%))	151 (46.32)	1142 (54.75)		
bFSH (U/L, ‾x ± *s*)	11.49 ± 5.89	10.55 ± 5.76	1.450	0.006
bE_2_ (pg/ml, ‾x ± *s*)	35.04 ± 17.10	34.66 ± 19.22	1.572	0.741
BMI (kg/m^2^, ‾x ± *s*)	23.79 ± 3.41	23.74 ± 3.56	2.853	0.814
AMH (ng/ml, M (P25, P75))	0.66 (0.32, 1.25)	0.73 (0.28, 1.43)	−0.283	0.812
Ovulation induction scheme				
Microstimulation (case (%))	227 (69.63)	1,429 (68.50)	0.167	0.683
Antagonists (case (%))	71 (21.78)	494 (23.68)	0.569	0.451
Natural cycle (case (%))	28 (8.59)	163 (7.81)	0.232	0.630
Abnormal semen in male^∗^ (case (%))	201 (61.66)	433 (20.76)	243.396	<0.01

^∗^Normal semen criteria: according to the WHO manual for the examination and processing of human semen (5th edition), semen was normal and there was no anti-sperm antibody. The details were as follows: concentration >15 × 10^6^/ml, total vitality >40%, premotor movement >32%, normal morphology >4%, and volume >1.5 ml. *P* < 0.05 was considered that the difference was statistically significant.

**Table 2:** Comparison of the clinical data and pregnancy outcomes between the ICSI group and IVF group when ≤3 eggs were retrieved.

Index	ICSI group (case) *n* = 326	IVF group (case) *n* = 2,086	*P* value
Gn time (d, ‾x ± *s*)	8.21 ± 3.13	8.43 ± 3.34	0.298
Total Gn (IU, ‾x ± *s*)	1,878.37 ± 1,001.69	1,854.62 ± 1,007.40	0.708
Number of eggs retrieved (x ± *s*)	1.94 ± 0.82	1.94 ± 0.82	0.997
MII rate (case (%))	543 (85.78)	3,467 (85.58)	0.895
2PN fertilization rate (case (%))	477 (87.85)	2,775 (80.04)	<0.01
Abnormal fertilization rate^∗^ (case (%))	66 (12.15)	692 (19.96)	<0.01
High-quality embryo rate (case (%))	258 (56.70)	1544 (56.74))	0.993
Cycle cancellation rate^∗∗^ (case (%))	27 (8.28)	256 (12.27)	0.037
Fresh embryo transfer			
Pregnancy rate (case (%))	30 (40.00)	178 (37.71)	0.705
Miscarriage rate (case (%))	4 (13.33)	27 (15.17)	0.794
Frozen-thawed embryo transfer			
Pregnancy rate (case (%))	89 (48.63)	128 (29.63)	<0.01
Miscarriage rate (case (%))	13 (14.61)	13 (10.16)	0.321
Cumulative pregnancy rate (case (%))	119 (46.12)	306 (33.85)	<0.01
Cumulative miscarriage rate (case (%))	17 (14.29)	40 (13.07)	0.742

^∗^(0PN + 1PN + multi-PN) fertilization. ^∗∗^Cancellation of cycles due to abnormal fertilization (multi-PN fertilization in the IVF group and 0PN + 1PN + multi-PN fertilization in the ICSI group).

**Table 3:** Comparison of the clinical data and pregnancy outcomes between ICSI and IVF groups when the number of retrieved eggs was one, two, and three, respectively.

Index	One egg retrieved		*P* value	Two eggs retrieved		*P* value	Three eggs retrieved		*P* value
	ICSI group	IVF group		ICSI group	IVF group		ICSI group	IVF group	
Number of case	119	774		107	660		100	652	
Gn time (d, ‾x ± *s*)	7.28 ± 3.67	7.77 ± 3.93	0.281	8.50 ± 2.75	8.59 ± 3.35	0.782	8.70 ± 2.84	8.87 ± 2.53	0.550
Total Gn (IU, ‾x ± *s*)	1,500.88 ± 1,109.45	1,590.79 ± 1,120.78	0.489	2,002.14 ± 924.42	1890.06 ± 978.93	0.273	2,069.28 ± 900.86	2,056.24 ± 867.90	0.889
MII rate (case (%))	116 (97.48)	663 (85.65)	<0.01	176 (82.24)	1,127 (85.37)	0.234	251 (83.67)	1,677 (85.74)	0.344
2PN fertilization rate (case (%))	100 (86.21)	498 (75.11)	0.009	147 (83.52)	904 (80.21)	0.301	230 (91.63)	1373 (81.87)	<0.01
Abnormal fertilization rate^∗^ (case (%))	16 (13.79)	165 (24.89)	0.009	29 (16.48)	223 (19.79)	0.301	21 (8.37)	304 (18.13)	<0.01
High-quality embryo rate (case (%))	47 (50.54)	279 (56.47)	0.290	75 (54.35)	501 (56.67)	0.608	136 (60.71)	764 (56.88)	0.284
Cycle cancellation rate^∗∗^ (case (%))	17 (14.29)	177 (22.87)	0.035	9 (8.41)	60 (9.09)	0.820	1 (1.00)	19 (2.91)	0.268
Fresh embryo transfer									
Pregnancy rate (case (%))	8 (44.44)	18 (21.43)	0.042	10 (40)	52 (37.41)	0.516	12 (37.50)	108 (43.37)	0.191
Miscarriage rate (case (%))	1/8 (12.5)	4/18 (22.22)		1/10 (10.0)	7/52 (13.46)		2/12 (16.67)	16/108 (14.81)	
Frozen-thawed embryo transfer									
Pregnancy rate (case (%))	27 (42.19)	52 (28.26)	0.039	30 (46.88)	38 (28.57)	0.011	32 (58.18)	38 (33.04)	0.002
Miscarriage rate (case (%))	2/27 (7.41)	4/52 (7.69)		6/30 (20)	5/38 (13.16)		5/32 (15.63)	4/38 (10.53)	
Cumulative pregnancy rate (case (%))	35 (42.68)	70 (26.12)	0.004	40 (44.94)	90 (33.09)	0.043	44 (50.57)	146 (40.11)	0.076
Cumulative miscarriage rate (case (%))	3/35 (8.57)	8/70 (11.43)	0.652	7/40 (17.5)	12/90 (13.33)	0.535	7/44 (15.91)	20/146 (13.70)	0.713

*P* < 0.05 was considered that the difference was statistically significant. ^∗^(0PN+ 1PN + multi-PN) fertilization. ^∗∗^Cancellation of cycles due to abnormal fertilization (multi-PN fertilization in the IVF group and 0PN + 1PN + multi-PN fertilization in the ICSI group).

## Data Availability

All the data generated or analyzed during this study are available from the corresponding author upon reasonable request.
